# Astragalus Polysaccharides/PVA Nanofiber Membranes Containing Astragaloside IV-Loaded Liposomes and Their Potential Use for Wound Healing

**DOI:** 10.1155/2022/9716271

**Published:** 2022-05-11

**Authors:** Yuan Yue, Xinjun Liu, Lan Pang, Yue Liu, Yuzhu Lin, Ting Xiang, Jie Li, Shiqin Liao, Yunlan Jiang

**Affiliations:** ^1^Chengdu University of Traditional Chinese Medicine, Chengdu, China; ^2^Hospital of Chengdu University of Traditional Chinese Medicine, Chengdu, China

## Abstract

Delayed wound healing is a common and serious complication in diabetic patients, especially the slow healing of foot ulcers, which seriously affects the quality of life of patients and is also the most important risk factor for lower limb amputation. The multifunctional novel dressing prepared by loading the polymer nanofibers with anti-inflammatory and prohealing plant extracts can promote the wound repair of these ulcers by electrospinning technology. Liposomes are nanoparticles prepared from phospholipids and have been widely used as drug delivery systems. Liposomes can be combined with electrospun nanofibrous webs to facilitate local and sustained delivery of loaded bioactive substances. In this study, liposomes were prepared with astragaloside IV (AS) by employing a modified ethanol injection method and conducting the physical and chemical characterization (e.g., the particle size, polydispersity index, zeta potential, and entrapment efficiency). Astragalus polysaccharides were extracted from *Astragalus membranaceus*. Subsequently, we prepared the electrospun polyvinyl alcohol (PVA)/astragalus polysaccharide (APS)/astragaloside IV (AS) nanofibers. The morphology of the produced ASL/APS/PVA, APS/PVA, and PVA nanofibers were analyzed by scanning electron microscopy (SEM), and it turns out that the addition of astragalus extract made the fiber diameter smaller and the fibers arranged neatly with no dripping. An induced diabetic rat model was built, and a diabetic ulcer model was built by total cortical resection to assess the prorepair ability of the prepared nanofibers. According to in vivo animal experiments, the nanofibrous membrane loaded with APS and ASL was reported to inhibit the occurrence of wound inflammation, enhance the deposition of collagen fibers (*P* < 0.05) and the repair of regenerated epithelium (*P* < 0.05), and effectively strengthen the wound healing of diabetic rats (*P* < 0.05). In brief, PVA-loaded APS/ASL nanofibrous membranes refer to a prominent wound healing dressing material, which can effectively facilitate the healing of diabetic wounds, and they are demonstrated to be highly promising for application in diabetic wound dressings and tissue engineering.

## 1. Introduction

Diabetes is accompanied by a number of complications, among which the skin wound-healing process refers to a major severe complication damaged by diabetic metabolism, vascular neuropathy, and inflammation, thereby causing wound-healing failure [1, 2]. Nearly 19%∼34% of diabetic patients will develop diabetic foot, and 20% of diabetic foot patients will suffer from amputation as impacted by different degrees of infection, which imposes huge economic burden on patients and the society [3–5]. Early and effective management of patients with diabetic foot can reduce the incidence of complications and prevent amputation and death. Debridement, reduction of infection, vascular reconstruction, and decompression remain the major principles for treating diabetic ulcer [6]. However, decreased endogenous growth factor level and activity in diabetic wound resulted in decreased collagen deposition and granulation tissue production, leading to poor wound treatment effect. However, it is noteworthy that modern clinical preparations are progressively derived from medicinal plants and have been widely used in ulcer and wound management. According to existing studies, the use of two herbal formulations reduced leg amputations in patients with diabetic ulcers by 85% [7]. This has inspired researchers to explore the potential wound-healing effects of medicinal plants and to isolate chemicals associated with wound healing.

*Astragalus membranaceus*, i.e., Huang Qi in China, a major herbal remedy for diabetic foot ulcers, has been exploited in traditional Chinese medicine (TCM) for hundreds of years. A Chinese herbal formula containing *Astragalus membranaceus* was reported to be able to significantly facilitate fibroblast proliferation (Hs27) and angiogenesis, and it was found to exhibit significant anti-inflammatory activity [8]. *Astragalus membranaceus* covers various bioactive components, among which the major pharmacological components facilitating wound healing include polysaccharides and saponins exhibiting immunomodulatory function and capable of stimulating cell metabolism [9]. APS and AS are the main aqueous extracts of *Astragalus membranaceus* and have pharmacological effects such as lowering blood glucose, promoting fibroblast proliferation, and cell growth factor expression in the treatment of diabetes and its complications [10, 11]. According to Zhao et al. [12], APS is capable of facilitating proliferation, migration, and cycle progression of fibroblasts, as well as promoting the reepithelialization, revascularization, and cytokine fluctuation of transforming growth factor (TGF)-*β*1, basic fibroblast growth factor (bFGF), and epidermal growth factor (EGF). Luo et al. [13] employed astragaloside IV into streptozotocin-induced diabetic mouse wound therapy, and they demonstrated that astragaloside IV is capable of facilitating collagen deposition and extracellular matrix (ECM)-related gene expression, as well as promoting wound tissue neovascularization and endothelial cell proliferation. However, the hydrophobicity of AS requires selection of suitable external drug carriers to expedite the release of drug action. Liposomes have microscopic phospholipid bubbles with a double membrane structure, good biocompatibility, and nanoscale size, which have aroused extensive attention as drug carriers. At present, considerable liposomes delivery systems with different functions have been developed [14, 15] and high efficacy has been achieved in local skin delivery [16]. Furthermore, when liposomes are combined with bioengineered scaffolds, the 3D structure of scaffolds is capable of increasing the therapeutic effects of liposomes [17].

Electrospinning is popular for preparing nonwoven mats, which have shown potential applications in a wide variety of fields, including wound dressing [18]. The nanofibers have unique properties and drug loading capability for promoting cell migration and adhesion and anti-infection ability [19]. Thus, they are good candidates for wound healing, particularly for diabetic foot wound care [20]. Yang et al. [21] loaded Astragalus polysaccharides into nanofiber pads for diabetic wound treatment which achieved good results and accelerated the rate of wound repair. He et al. [22] electrospinned polycaprolactone and quaternized chitosan-graft-polyaniline polymer solutions to prepare a series of nanofiber membranes with antibacterial, antioxidant, and electroactive properties, confirming that the nanofibers can promote wound collagen deposition, granulation tissue proliferation, and angiogenesis. However, most of those nanofiber mats were prepared by a binding solution containing drugs and polymers. The electrospinning is developing along three directions; one is the large-scale production of new polymer nanofibers [23], the second is the multiple-fluid electrospinning for creating core shell [24], Janus [25], trilayer core shell [26], and other complicated nanostructures [27], and the third is the combination of electrospinning with other traditional techniques [28]. In this study, we combined liposomes prepared by ethanol infusion with electrospinning for the fabrication of novel wound dressings.

Polyvinyl alcohol (PVA) refers to a synthetic polymer, which is highly biocompatible in vivo with nontoxic property. For its hydrophilic and porous structure properties, it is extensively applied to investigate medical biomaterials and tissue regeneration [29]. Thus far, numerous studies in biomedicine have combined polymers with plant extracts to achieve nanoelectrospinning [30–33]. Saeed et al. used turmeric extract mixed with PVA on rat wounds and showed effective wound-healing ability [34]. Mwiiri et al. [35] successfully developed PVA-based electrospun nanofibers by mixing different molecular weights and concentrations of PVA with birch integument extracts, showing high antibacterial activity and biocompatibility.

Thus, this study fabricated three electrospun nanofiber (NF) membranes, ASL/APS/PVA, APS/PVA, and PVA nanofibrous membranes, with the use of PVA as the polymer matrix and APS and ASL as the carriers through electrospinning (Figure 1). Next, they were administered to a skin wound based on a diabetic rat model. The wound-healing processes were assessed based on hematoxylin-eosin (HE) and Masson staining for inflammatory reaction and collagen synthesis and through macroscopic observation of wound closure.

## 2. Materials and Methods

### 2.1. Materials

In this study, APS (purity >80%) was extracted from the laboratory. Chengdu Pharmaceutical Market, China (Chengdu, China), offered SR. Chengdu Lemeitian Pharmaceutical Technology Co., Ltd. (Chengdu, China) provided astragaloside IV with >99.8% purity. Chengdu Kelong Chemical Reagent Factory (Chengdu, China) offered PVA. Aladdin (Shanghai, China) offered streptozotocin (STZ) and cholesterol (purity >95%). AVT Pharmaceutical Tech Co., Ltd. (Shanghai, China) provided egg yolk lecithin. Shenzhen Reward Life Tech Co., Ltd. (Shenzhen, China) provided isoflurane. Chengdu Koen Experimental Equipment Co., Ltd. (Chengdu, China) offered absolute ethanol, diethyl ether, and acetone. Sinopharm Chemical Reagent Co., Ltd.(Shanghai, China) offered neutral gum, xylene, and ethanol. Servicebio (Wuhan, China) provided the HE dye solution set and the Masson dye solution set.

### 2.2. Extraction of Astragalus Polysaccharide

We extracted APS from AR by water extraction and alcohol precipitation [36]. 200 g of *Astragalus membranaceus* was added to 95% ethanol (1 L) and petroleum ether (1.2 L) for reflux for 2 h, respectively, and it was repeated twice to remove fat-soluble substances and then extracted with boiling water (2 L) for 2 h. The extraction process was repeated twice, and the extracts were integrated, filtered, and concentrated to 1/3. Next, the protein was deproteinized with Sevag reagent [37], and anhydrous ethanol (4 times) was added and stirred efficiently and then precipitated for 12 h. Lastly, the precipitate was collected, washed with anhydrous ethanol, ether, and acetone, and dried in vacuum to produce astragalus polysaccharide. Finally, the phenol-sulfuric acid method was used to determine polysaccharide content [38].

### 2.3. Preparation of ASL

Liposomes were produced based on the modified ethanol injection approach. To be specific, cholesterol, lecithin, and AS were dissolved in 2 ml of ethanol solution and then instilled dropwise into 10 ml of pure water with a magnetic stirrer for 2 h to solidify nanoparticles in cold water. Furthermore, ASL was produced by passing through a 0.45 *μ*m microporous filter membrane after the anhydrous ethanol was volatilized.

### 2.4. Assessment of ASL

#### 2.4.1. Particle Size Analysis and Zeta Potential Measurement

We diluted liposomes with double-distilled water. Next, the conductivity was regulated to 50 ms/cm with sodium chloride. Using the Helmholtz–Smoluchowski equation, the examined electrophoretic mobility was transformed into zeta potential. The mentioned process was carried out based on the software covered within the system.

#### 2.4.2. Encapsulation Efficiency (EE) and Drug Loading

The lipids preparation was dissolved in formaldehyde and subsequently spun for extracting the drug from the agent. The sample was centrifuged at 10,000 revolutions per minute for 10 min. The solution supernatant was extracted and diluted by using methanol, and drug concentration was ascertained based on high-performance liquid chromatography. The drug loading in ASL was ascertained based on the centrifugal method.

#### 2.4.3. Morphological Observation and Analysis by TEM

ALS was diluted with deionized water, and 10 *μ*l solution was dripped onto a 300-mesh copper wire. After 10 min, a nitrogen blowing instrument was employed for drying the ASL. 2% phosphotungstic acid was used for staining for 10 min, and the excess phosphotungstic acid was drawn; the nanosome morphology was characterized through electron microscope projection.

### 2.5. Preparation of the Electrospun Solutions

PVA spinning solution (9%, w/v) was prepared by dissolving 0.9 g PVA in 10 ml pure water and stirring for 4 h. 0.1 g APS was weighed and then introduced to 2 ml pure water, and 0.9 g PVA was weighed and dissolved in 8 ml pure water. The solution was stirred for 4 h first and then mixed and stirred for 4 h. Lastly, 0.9 g PVA and 0.1 g APS were weighed and dissolved in the prepared astragaloside liposome solution (2 ml) to produce ASL/APS/PVA spinning solution.

### 2.6. Electrospinning of the Blend Solution

Three electrospinning solutions were electrospun with an electrospinning machine (TL-QX-01, Tong Li Tech Co., Ltd, Shenzhen, China). The loading was achieved for the solution through a 20 ml plastic syringe with a 20-gauge stainless steel needle attached as a nozzle. The voltage was 21 kV, the nozzle speed was 0.4 ml/h, and the receiving distance was 12 cm.

### 2.7. Fiber Topography Characterization

The resulting nanofibers' morphology was characterized and photographed by a scanning electron microscope. Three fiber pictures were randomly selected, the diameter of the prepared nanofiber mats was measured using Image J software, and this study determined the average diameter.

### 2.8. Repair Effect of the Nanofiber Membrane on Skin Wound in Diabetic Rats

Chengdu Dashuo Laboratory Animal Co., Ltd. provided SD rats aged 8 weeks. The rats were housed at constant temperature (25 ± 1°C) and accessed normal diet and water freely, and bedding was changed per day. The experimental operations were overall consistent with the Guidelines for the Management of Laboratory Animals of Chengdu University of Traditional Chinese Medicine. All animal experiment procedures were in accordance with the Chengdu University of Traditional Chinese Medicine Animal Welfare Guidelines (Animal Experiment Ethics Approval Number: 2014 DL-023). Establishment of the diabetic rat model: 16 SD rats weighing 180∼220 g randomly fell into 4 groups, with 4 rats in the respective group. After fasting for 12 h, STZ sodium citrate buffer (pH 4.3) was intraperitoneally injected at a concentration of 45 mg/kg. The blood glucose concentration was measured once 3 days after modeling. The automatic blood glucose meter (Roche Diabetes Care GmbH, Shanghai, China) was used. The blood glucose exceeded 16.7 mmol/L, thereby demonstrating the successful modeling. Otherwise, additional STZ continued. All rats underwent wound model preparation after inhalation of isoflurane gas anesthesia, and the hair on the back of the rats was removed by hair removal cream. Moreover, to create six full-thickness skin wounds of nearly 0.8 cm in diameter, the holes were made on both sides of the spine. The wounds were covered with ASL/APS/PVA, APS/PVA, and PVA nanofibers, and the naturally healed wounds acted as the control (NH group), and the back wounds of rats were wrapped with gauze to prevent dressings and they were housed in single cages.

### 2.9. Wound-Healing Studies

Macroscopically, the skin healing of the respective group was identified at 3, 7, 11, and 15 days after the surgery. The wounds of the respective group were photographed, and the wound-healing area of the respective group at different time points was calculated with Image J software. The extent of wound healing is expressed as the percentage, i.e., the wound size (%) = [(*W*_0_ − *W*_*n*_/*W*_0_] × 100%, where *W*_0_ and *W*_*n*_ represent the exposed areas of the wounds on days 0 and 3, 7, 11, and 15, respectively.

### 2.10. Histological Examination

Wound new tissues from the experimental group at the respective time point were taken, frozen, sectioned, fixed in 4% paraformaldehyde, stained by using HE and Masson, and then characterized by employing a light microscope. HE staining: paraffin sections were dewaxed to water, which include xylene treatment, gradient alcohol dehydration, and water washing. Hematoxylin dyeing: hematoxylin dyeing solution was dyed for 3–5 min, cleaned with tap water, differenciated with the differentiation solution, washed washing with tap water, returned to bule color with the blue return solution, and rinsed with water. Eosin dyeing: gradient alcohol dehydration, eosin dyeing solution. The dehydrated sheet comprised gradient alcohol dehydrated, xylene transparent, and neutral gum seal sheet. Masson staining: paraffin sections were dewaxed to water, which include xylene treatment, fractional ethanol dehydration, and tap water washing. Being soaked in Masson A overnight and then washed with running water. Being sectioned into Masson B and Masson solution C equal ratio mixture of the dye, soaked, washed with tap water, subjected to alcohol differentiation with 1% hydrochloric acid, then washed with tap water being soaked in Masson D solution and rinsed with tap water. Being soaked in Masson E solution. Being drained and soaked in Masson F solution. Being rinsed and differentiated with 1% glacial acetic acid and dehydrated with anhydrous ethanol. Being placed into the third cylinder of anhydrous ethanol for 5 min, xylene transparent, and neutral gum sealed sheet. The stained slices were observed under an upright optical microscope (Nikon, Japan).

### 2.11. Statistical Methods

The data were processed with SPSS 21.0 statistical software, and continuous variables were statistically expressed as mean ± standard deviation. Means between multiple groups were compared using multivariate ANOVA and between two groups by performing the LSD test. *P* < 0.05 was considered to be statistically significant.

## 3. Results

### 3.1. ASL Characteristics Analysis

In this study, astragaloside IV binds with egg yolk lecithin and cholesterol to form astragaloside IV liposomes. Average particle size and zeta potential are capable of predicting the stability of liposome nanoparticles, i.e., the characteristics of traditional Chinese medicine. Particles with high zeta potential are less likely to aggregate due to electrical repulsion. According to Figure 2, nanoparticles' morphology and surface state examined by TEM are presented. In Figure 2(a), the liposomes could be observed to have a spherical shape under an electron microscope.  Figure 2(b) shows that the particle size of the prepared liposomes was (143.23 ± 3.25) nm and PDI was 0.11 ± 0.048. The zeta potential and DEE are presented in Table 1. The zeta potential was (−11.2 ± 1.35) mV, EE value was 89 ± 6 %, and drug loading was 85 ± 3%, indicating that the liposomes were uniformly dispersed, not easy to produce aggregation phenomenon, the size met the requirements.

### 3.2. Characterization of Electrospun Nanofibers

The surface morphologies of ASL/APS/PVA, APS/PVA, and PVA nanofiber membranes were observed by SEM, as presented in the scanning electron micrographs (Figure 3). The three nanofibers had smooth surfaces with uniform thicknesses and no droplets, and adhesion and bifurcation phenomena were found on the surfaces. Besides, the surfaces were randomly arranged, with (210.56 ± 91.303) nm, (138.679 ± 93.616) nm, and (145.68 ± 66.856) nm diameters, respectively, and no significant difference was identified in the diameter of the three fiber groups (*P* > 0.05).

### 3.3. Observation of Wound Healing

Figure 4(a) presents the gross observation of the wound area in various healing time periods in terms of diabetic mice wound: untreated (Blank), diabetic mice wound treated with PVA nanofibrous membranes, diabetic mice wound treated with APS/PVA nanofibrous membranes, and diabetic mice wound treated with ASL/APS/PVA nanofibrous membranes. A few days after the surgery, the wound gauze had basically fallen off. The wound healing area took up 65.3 ± 17.4%, 81.1 ± 12.3%, 83.8 ± 11.9%, and 94.5 ± 6.1% in the Blank, PVA nanofibrous membranes, APS/PVA nanofibrous membranes, and ASL/APS/PVA nanofibrous membrane groups (Figure 4(b)), respectively. On the 7th day after operation, compared with the negative control, the wound area of all fibrous membrane groups was significantly reduced. The wound of the ASL/APS/PVA nanofibrous membrane group achieved large area healing, basal congestion at the center of the wound, massive granulation tissue proliferation, and no infection. As opposed to the mentioned statement, although the APS/PVA nanofibrous membrane group healed faster than the negative control and PVA nanofibrous membranes alone group, its healing was slower than the ASL/APS/PVA nanofibrous membrane group, with less granulation tissue, thereby demonstrating that the addition of ASL, in comparison with APS nanofibrous membrane alone, could facilitate wound healing. On the 15th day after the operation, considerable collagen fibers and a small number of fibroblasts were found in the dermis of the new skin of the wound in the ASL/APS/PVA nanofibrous membrane group and obvious skin appendages were reported in the differentiation stage. The epidermal layer structure was consistent with the normal skin epidermal structure. Moreover, the wound healing rate rose significantly in the APS/PVA nanofibrous membrane group compared with the control group of PVA nanofibrous membranes alone, whereas the epidermis and dermis remained in the repair state and the wound was not closed overall. The healing rate of the group with PVA nanofibrous membranes alone was slower, whereas the wound healing rate reached over that of the negative control, probably due to the characteristics exhibited by the extracellular matrix of the nanofibrous membrane and the three-dimensional network structure. As a result, wound secretions could be absorbed, cell adhesion and migration could be facilitated, and the repair of tissue wounds could be improved.

### 3.4. Histological Staining

Figure 5 illustrates the results of HE-stained tissue sections and analyzes the wound structure in the healing process in the respective experimental group. At 3 days, distinct dark blue cell clusters were found in all groups, thereby indicating the production and accumulation of neutrophils. At 11 days, the ASL/APS/PVA nanofibrous membrane group had significantly reduced neutrophils, diminished inflammation, more neovascularization, and increased granulation tissue. Slight inflammatory cell infiltration was identified in the APS/PVA and PVA nanofibrous membrane groups, while significant neutrophil accumulation was identified in the blank group, and there was still a significant inflammatory response. There was always inflammation in the whole healing process of the blank group, which was significantly higher than that of the PVA nanofibrous membrane group. As opposed to the mentioned statement, minimal inflammation was identified at 7 days in APS/PVA and ASL/APS/PVA nanofibrous membrane groups, which was a response in the normal healing process, and no signs of inflammation were found at 11 and 15 days. The mentioned observations indicated that APS/PVA and ASL/APS/PVA nanofibrous membranes could significantly reduce the inflammatory response of the wound surface. At 15 days, the regenerated epithelial tissues of the wounds treated in the APS/PVA and ASL/APS/PVA nanofibrous membrane groups had been completely covered, and the stratum corneum and basal layer were intact, while the epithelial tissues in the blank group remained in the repair state and formed no epithelialization and partial epithelialization was identified in the PVA nanofibrous membrane group. As indicated from the Masson staining of wound tissue (Figure 6), the more gel blue staining area, the deeper the staining and the thicker the fibril deposition; according to PVA, APS/PVA, and ASL/APS/PVA nanofibrous membrane groups, the gel blue staining area was more, and deep staining, fibril deposition was thicker, and APS/PVA and ASL/APS/PVA nanofibrous membrane groups were most obvious, of which ASL/APS/PVA nanofibrous membrane group's collagen fiber deposition was the most closely arranged. However, collagen fibers were disorganized and deposited less in the blank group. The mentioned results demonstrated that the electrospun nanofiber membrane could facilitate the tissue repair of diabetic ulcer tissue.

## 4. Discussion

Diabetes refers to a major and significant challenge faced by clinical medicine worldwide, and the incidence of chronic skin ulcers is rising as well. According to the existing reports, there are about 91–26.1 million new patients with diabetic foot ulcers each year [3], which has a high incidence, while seriously reducing the quality of life and psychosocial adaptability of patients [39]. Electrospinning technology is being extensively applied in the biomedical field to produce polymer nanofibers for treating wounds, burns, and diabetic ulcers [40]. To facilitate the repair of diabetic wounds, various cells, growth active factors, and drugs have been embedded in TEMS (e.g., hematopoietic stem cells [41], insulin [42], and doxycycline [43]), whereas the activity of the mentioned cells and biological macromolecules is difficult to maintain. In this study, APS and AS, with established effects on facilitating fibroblast growth and endothelial protection, were loaded to nanofibers by electrospinning and applied to the wounds of diabetic rats to assess their effects on tissue repair.

The treatment mode based on combination drugs revealed the synergistic advantage of drug combination, which is termed “compound” in TCM. On the whole, this synergism indicates the effect exerted when ≥2 drugs were used in combination was greater than that when the respective drug acted alone. APS and astragaloside IV could protect vascular endothelial cells and facilitate angiogenesis. The poor solubility of astragaloside IV in water and the low oral bioavailability limit the effect of astragaloside IV. Liposomes are vesicle structures with hydrophilic ends in both inner and outer layers and a hydrophobic interlayer in the middle. Biocompatibility can encapsulate both water-soluble drugs and water-insoluble drugs. Therefore, in this study, astragaloside IV was encapsulated into liposomes. However, there are some problems in the application of liposomes, such as the lack of three-dimensional structure and the difficulty in maintaining a matching dose at the injury site. Electrospun nanofibers are widely used as drug carriers in many biomedical applications due to their high specific surface area, high porosity, small size effect, and surface effect. In this study, astragaloside IV-encapsulated liposomes were loaded into PVA nanofibers and liposome-loaded electrospun fiber scaffolds were successfully prepared, which not only increased the hydrophilicity and stability of astragaloside IV but also achieved sustained-release drug delivery and prolonged the action time. Future studies can further explore whether liposomes are present in PVA nanofibers in a holistic manner. Astragalus polysaccharides and astragaloside IV liposomes were mixed with PVA to make drug-loaded nanofibers through electrospinning to determine their effects on tissue regeneration in diabetic wounds. The structure of nanofibers was found based on scanning electron microscopy, and the addition of APS and astragaloside nanoparticles reduced the diameter of nanofibrous membranes, probably due to the decrease in the viscosity of the spinning solution.

This study adopted a common animal model of STZ-induced diabetic skin wounds and used acute full-thickness skin injury to replace spontaneous diabetic skin ulcers. We took out the wound surface and made macroscopic observation and histological examination on the wound surface. As revealed from the results, compared with the blank group, the 15-day nanofiber membrane could hinder the inflammatory response, facilitate collagen deposition and epithelial tissue production, and positively impact the healing of diabetic wounds, while the ASL/APS/PVA nanofibrous membrane group had the optimal wound repair effect, which showed an association with the promotion of APS and AS on wound healing and also verified that the synergistic effect of the two by electrospinning technique was better than that by using Astragalus polysaccharide alone. Furthermore, HE staining revealed that the reepithelialization rate of ASL/APS/PVA and APS/PVA nanofibrous membrane groups was significantly faster than that of other groups, and the inflammatory response was significantly lower than that of other groups. According to Masson's trichrome staining, the treatment of nanofibrous membranes significantly increased the deposition of nanofibrous membranes in diabetic wounds, which is critical to enhancing wound healing effects and facilitating functional recovery [44].

## 5. Conclusion

This study employed electrospinning technology to prepare PVA, APS/PVA, and ASL/APS/PVA nanofibers membranes, which were applied to the wounds of full-thickness skin defects in diabetic rats. The synergistic effect of APS and AS in nanofiber membranes exceeded that of APS alone, which could inhibit inflammation, facilitate collagen deposition and wound reepithelialization better, and positively impact diabetic wounds. As revealed from the results, the nanofiber membrane containing APS and AS could be a worthwhile method for treating diabetic wounds, and subsequent research can also pay more attention to the synergistic effect of traditional Chinese medicine.

## Figures and Tables

**Figure 1:** Schematic diagram of preparation and application of nanofibers.

**Figure 2:** TEM observation (a) of astragaloside IV-loaded ASL. Size distribution (b) of astragaloside IV-loaded ASL.

**Figure 3:** SEM images of the PVA (a), APS/PVA (c), and ASL/APS/PVA (e) electrospun nanofiber membranes and their diameter distribution illustration (b, d, f).

**Figure 4:** Photographic images of wound healing (a). Graphical illustration of the changes in wound size (b) on days 3, 7, 11, and 15 for the developed nanofibrous dressings of ASL/APS/PVA, APS/PVA, PVA, and the untreated negative control (^*∗*^*P* < 0.05 versus PVA).

**Figure 5:** (a) Representative HE images of groups Blank, PVA, APS/PVA, and ASL/APS/PVA at days 3, 7, 11, and 15. (b, c) Graphical representation of the regenerated skin tissues in the four groups at days 7and 15 after operation. All images magnification: ×200; scale bars: 100 *μ*m (^*∗*^*P* < 0.05, versus PVA).

**Figure 6:** (a) Micrographs of Masson-stained tissues of wounds treated with PVA, APS/PVA, and ASL/APS/PVA and untreated negative control at days 3, 7, 11, and 15. (b, c) Graphic representation of collagen fibers in the healing process within four groups. All images magnification: ×200; scale bars: 100 *μ*m (^*∗*^*P* < 0.05, versus PVA).

**Table 1:** Characteristics of ASL.

Sample	Particle size (nm)	Zeta potential (mV)	DLE (%)	PDI	EE (%)

ASL	143.23 ± 3.25	−11.2 ± 1.35	4.19 ± 0.66	0.11 ± 0.048	89 ± 6

Abbreviations: DLE, drug loading efficiency; PDI, polydispersion index; EE, encapsulation efficiency. Data are expressed as mean ± SD.

## Data Availability

The experimental data used to support the findings of this study are included within the article.
